The article "miR-219-5p targets TBXT and inhibits breast cancer cell EMT and cell migration and invasion" was retracted in 2024. Reasons: duplicated images; overlap with earlier publications; unreliable data; concerns about the data.

# miR-219-5p targets TBXT and inhibits breast cancer cell EMT and cell migration and invasion

**DOI:** 10.1042/BSR20210318

**Published:** 2021-08-12

**Authors:** Qin Ye, Xing Wang, Mei Yuan, Shuaishuai Cui, Yuanyuan Chen, Zhaodi Hu, Dandan Liu, Conghui Han, Bibo Li, Dahu Chen

**Affiliations:** 1 School of Life Sciences, Jiangsu Normal University, Xuzhou 221116, China; 2 School of Life Sciences, Shandong University of Technology, Zibo 225000, China; 3 Department of Urology, Xuzhou Central Hospital, Xuzhou 221009, China; 4 Department of Urology, Taizhou Hospital Affiliated to Nanjing University of Chinese Medicine, Taizhou 225300, China

**Keywords:** cell invasion, cell migration, EMT, miRNA, TBXT

## Abstract

miR-219-5p has been reported to act as either a tumor suppressor or a tumor promoter in different cancers by targeting different genes. In the present study, we demonstrated that miR-219-5p negatively regulated the expression of TBXT, a known epithelial–mesenchymal transition (EMT) inducer, by directly binding to TBXT 3′-untranslated region. As a result of its inhibition on TBXT expression, miR-219-5p suppressed EMT and cell migration and invasion in breast cancer cells. The re-introduction of TBXT in miR-219-5p overexpressing cells decreased the inhibitory effects of miR-219 on EMT and cell migration and invasion. Moreover, miR-219-5p decreased breast cancer stem cell (CSC) marker genes expression and reduced the mammosphere forming capability of cells. Overall, our study highlighted that TBXT is a novel target of miR-219-5p. By suppressing TBXT, miR-219-5p plays an important role in EMT and cell migration and invasion of breast cancer cells.

## Introduction

Although much progress has been made in cancer research, breast cancer remains a major public health concern, as it is the most diagnosed cancer in women worldwide and the second leading cause of cancer-related deaths [1,2]. Breast cancer initiates as a local disease but it often metastasizes to many other important organs, which is the main cause of breast cancer-related deaths [3]. The current treatment strategies, including surgery, chemotherapy and radiation therapy, control many localized breast tumors very well but have no effectiveness on containing the development of breast cancer metastasis. Thus, identifying novel molecular markers that can serve as appropriate therapeutic targets for more effectively controlling and treating breast cancer metastasis is an urgent task.

The metastatic cascade is a multistep process in which tumor cells, by changing their genetic and epigenetic characteristics, can survive in the new site that is distant from the original tumor site. It has been indicated that the epithelial–mesenchymal transition (EMT) is the main mechanism underlying the invasiveness and metastasis of various cancers [4,5]. The EMT is an evolutionally conserved program that is involved in developmental, physiological and pathological processes. During the EMT process, epithelial cells lose their cell–cell adhesion feature and cell polarity, and acquire migratory and invasive properties to convert into mesenchymal cells. This transition and new cell characteristics are indispensable not only for many developmental processes but also for the initiation of metastasis of cancer progression. Cell invasion is necessary for the initiation of metastasis and is enabled by EMT. It has been known that transcription factors [6,7], growth factors [8], extracellular ligands [9], epigenetic modulations [10] and microRNAs (miRNAs) [11–15] participate in regulating EMT process.

TBXT encodes an embryonic nuclear transcription factor that binds to a specific DNA element, the palindromic T-site. It binds through a region in its N-terminus, called the T-box [16], and affects transcription of genes required for mesoderm formation and differentiation [17]. The target genes regulated by TBXT in different species include those playing important roles in cell movement, cell shaping and cell–cell adhesion. There have been many studies on the function of TBXT in mice and zebrafish [17,18]. In vertebrates, TBXT participates in the regulation of the progenitors and their differentiated descendants [16–19]. TBXT is also overexpressed in a range of human carcinomas [20,21], where it regulates epithelial tumor plasticity by inducing epithelial tumor cells to undergo the EMT [22], which often contributes to the metastasis of tumor cells [23,24].

Because of the essential roles of TBXT in early development and in cancer progression, it is crucial to understand how its expression is regulated. There are some reports regarding the regulation of TBXT expression. For example, *Xbra*, an ortholog of TBXT in *Xenopus*, can be induced by members of the fibroblast growth factor [25] and transforming growth factor-β (TGF-β) families, such as activin [26], and repressed by Goosecoid and Mix.1 [27]. However, to the best of our knowledge, the mechanisms of controlling TBXT expression are not well understood.

miRNAs play important roles in gene expression regulation in mammals. They are evolutionally conserved small non-coding RNAs that typically comprise 18–25 nucleotides and are widely expressed in mammalian cells. By binding to the 3′-untranslated region (3′-UTR) of target mRNAs, miRNAs trigger either cleavage or translation inhibition of their target mRNAs [28]. miRNAs are involved in many cellular processes such as proliferation, development, differentiation, apoptosis and carcinogenesis. In terms of cancer, miRNAs can function either as a tumor suppressor or as a tumor promoter, whcih depends on their tissue-specific expression patterns and their mRNA targets [29]. Although there has been a great deal of studies on the roles of miRNAs in EMT and cancer metastasis [14], few have focused on effects of miRNA on regulation of TBXT, an important EMT inducer and metastasis promoter in breast cancer.

In the present study, we showed that TBXT is a novel target of miR-219-5p. Through inhibiting TBXT, miR-219-5p represses breast cancer cell EMT, migration and invasion *in vitro* and decreases cancer stem cell (CSC) features of breast cancer cells.

## Materials and methods

### Cell culture

HEK293T, MDA-MB-231, MCF-7 and BT474 cells were cultured in DMEM (high glucose) supplemented with 10% fetal calf serum, 100 U/ml of antibiotics including penicillin and streptomycin. MCF-10A cells were cultured in DMEM/F12 supplemented with 5% horse serum, EGF (20 ng/ml), hydrocortisone (0.5 mg/ml), cholera toxin (100 ng/ml), insulin (10 μg/ml) and 100 U/ml antibiotics including penicillin and streptomycin. Cells were housed in humidified 5% CO_2_ incubator at 37°C.

### Cell viability assay

Cell viability assay was determined by using LDH Cytotoxicity Detection Kit (Takara, MK401) and was performed following the protocol of manufacturer.

### Plasmids and short hairpin RNA

pBabe-puro retroviral vector was used to clone human miR-219 precursor sequences that were PCR amplified from normal genomic DNA. Primers for miR-219-5p precursor cloning are: F: 5′-ATGCGGATCCCTTCCCAATGGGAGCTCCATC-3′; R: 5′-ATGCGAATTCTTCTCAGGACTAGAAGGCTA-3′. A TBXT UTR fragment was cloned into the pMIR-REPORT luciferase construct, using the following primers: F: 5′-TAGCACTAGTGTAAACTCCACCAGTCCTACTTT-3′; R: 5′-TAGCAAGCTTGGCTTCACTAATAACTGGACGA-3′. The human TBXT open reading frame (ORF) expression plasmid, miR-219-5p inhibitor (HmiR-AN0330-AM03) and control plasmid (CmiR-AN0001-AM03-B) were purchased from Genecopia. The TBXT UTR mutant was generated using a QuikChange Site-Directed Mutagenesis Kit (Stratagene, San Diego, U.S.A.). Mutation primers: F: 5′-AGTAGCCAAActgAATCAGCAGAAAGCATTTTC-3′; and R: 5′-TTGTCAAAAGAAAAATATGAAACAG-3′.

### RNA isolation and real-time quantitative-PCR

RNA was isolated from cultured cells using TRIzol reagent. miRNA was extracted according to the manufacturer’s instructions using the miRVANA Kit (Ambion, Carlsbad, MA). miR-219-5p quantitative PCR (qPCR) was performed using the MystiCq® MicroRNA qPCR Assay Primer (MIRAP00276; Sigma, U.S.A.) and MystiCq® microRNA qPCR Control Primer (MIRCP00001; Sigma, U.S.A.). qPCR was conducted according to the manufacturer’s instructions. The primer sequences for qPCR analysis are as follows:

Nanog: F: 5′-GTCTTCTGCTGAGATGCCTCACA-3′;
  R: 5′-CTTCTGCGTCACACcATTGCTAT3-3′.
Aldh1: F: 5′-CTGCTGGCGACAATGGAGT-3′;
  R: 5′-GTCAGCCCAACCTGCACAG-3′.
TBXT: F: 5′-TATGAGCCTCGAATCCACATAGT-3′;
  R: 5′- CCTCGTTCTGATAAGCAGTCAC-3′.
18S RNA: F: 5′-TGTGCCGCTAGAGGTGAAATT-3′;
  R: 5′-TGGCAAATGCTTTCGCTTT-3′.

The qRT-PCR data analysis was performed by using the comparative *C*_t_ (2^−dd*C*_t_^) method. 18sRNA or U6 RNA was used as an internal control gene to normalize the amount of RNA or miRNA added to the first-strand cDNA synthesis reactions. The difference between the threshold cycle (*C*_t_) of the target gene and the *C*_t_ of the reference gene (18sRNA or U6) of the same sample was calculated as d*C*_t_. The difference of d*C*_t_ between treated cells and control cells was calculated as dd*C*_t_. The final quantitation result is presented as the fold change of target gene expression in treated cells relative to control cells, normalized to 18sRNA or U6 RNA.

### miRNA target analysis

TargetScan and miRBase programs were used to predict the genes that contain miR-219-5p binding site(s) in UTR sequence.

### Migration and invasion assays

Transwell migration and Matrigel invasion assays were performed as previously described [30]. The transwell system (Corning, New York, U.S.A.) was used for assays. Briefly, the cells supplemented with serum-free medium were respectively seeded into the upper chambers coated with (for invasion) or without (for migration) Matrigel. The lower chambers contained 500 μl of culture medium plus 10% FBS. After incubation for 48 h, cells on the upper chamber side of the membrane were scraped off with cotton swabs. The migrated or invaded cells were fixed with 70% ethanol, stained with 0.5% Crystal Violet. The cells on the lower side of the membrane were observed under microscope and at least five pictures were taken from each membrane randomly. The stained cells were manually counted from the pictures.

### Mammosphere assay

The mammosphere assay was performed according to the vendor’s (Stemcell Technologies, Vancouver, Canada) protocol. Briefly, single cell suspensions were seeded in the six-well ultra-low attachment plate (Corning, New York, NY, U.S.A.) at a density of 3.5–4.0 × 10^4^ cells in 2 ml of freshly prepared Complete MammoCult Medium (StemCell Technologies) per well. After incubation for 7 days, the number of mammospheres that were larger than 40 mm in diameter was counted.

### Luciferase reporter assay

Dual luciferase reporter assays were performed according to the manufacturer’s instructions (Promega, Madison, U.S.A.).

### Immunoblotting

Cell lysis and Western blot analysis were performed using standard methods. The following antibodies were used: anti-E-cadherin (SC-8426; Santa Cruz Biotechnology, Dallas, TX, U.S.A.), anti-N-cadherin (SC-271386; Santa Cruz), anti-vimentin (SC-6260; Santa Cruz), anti-Nanog antibody (SC-376915; Santa Cruz) and anti-β-actin antibody (610182; Sigma).

### Statistical analysis

Unless otherwise noted, each sample was assayed in triplicate (three separate cell cultures or three independent transfections). Cell viability and migration/invasion assays were repeated three to four times. The *in vitro* biochemical and molecular biological experiments were repeated three times. Unless otherwise noted, data were presented as the mean ± s.e.m., and the two-tailed Student’s *t* test was used to compare two groups. The differences were considered statistically significant when the *P*-values were <0.05.

## Results

### TBXT is a novel target of miR-219-5p and its expression is inhibited by miR-291-5p in breast cancer cells

To identify the miRNA that regulates TBXT, we used two computational algorithms, TargetScan and miRBase, to search for the regulatory miRNA for TBXT. MiR-219-5p was predicted to be a possible miRNA that regulates TBXT. TBXT mRNA contains a conserved miR-219-5p binding site in its 3′-UTR (Figure 1A). To verify this prediction, we subcloned the wildtype or mutant of TBXT 3′-UTR into a luciferase reporter vector. The ectopic expression of miR-219-5p reduced the activity of a luciferase reporter fused to wildtype TBXT 3′-UTR but not the activity of a reporter fused to a mutant TBXT 3′-UTR with mutations in the miR-219-5p seed-pairing region (Figure 1B). The results indicated that miR-219-5 p can directly bind to the 3′-UTR of TBXT and the observed down-regulation of luciferase activity by miR-219-5p directly depends on a single binding site in the TBXT 3′-UTR. We ectopically expressed miR-219-5p in MDA-MB-231 cells (Figure 1C) and found a pronounced reduction in TBXT mRNA level (Figure 1D) and protein level (Figure 1E) compared with mock cells. To further confirm the regulation of miR-219-5p on TBXT, we transfected MDA-MB-231 cells with miR-219-5p inhibitor and checked the expression of TBXT by qPCR in those cells. The miR-219-5p knockdown effect was shown in Figure 1F. We found that TBXT expression increased with the decreased expression of miR-219-5p (Figure 1G). These results indicated that TBXT is a novel target of miR-219-5p and the expression of TBXT is inhibited by miR-219-5p in breast cancer cells. Moreover, we performed qPCRs for miR-219-5p and TBXT in several different breast cancer cells and found that there is a negative correlation between miR-219-5p and TBXT expression in those cells (Figure 1H,I).

**Figure 1:** TBXT is a novel target of miR-219-5p (**A**) Partial sequence of human TBXT UTR containing miR-219-5p binding site; sequence of mature miR-219-5p; partial sequence of the generated mutant UTR of human TBXT in complementary sites for seed regions in miR-219-5p. (**B**) Relative luciferase activity of the luciferase reporter gene that a human TBXT 3′-UTR fragment containing the wildtype miR-219-5p binding sequence (WILD) or the mutant miR-219-5p binding sequence (MUTANT) was cloned downstream of it. The luciferase activity was analyzed in 293 T cells that were transfected with either miR-219-5p or the control vector (mock). The data are presented as means ± SD of three independent experiments, and statistical significance was determined by two-tailed, unpaired Student’s *t* test. (**C**) The expression level of miR-219-5p in mock cells and miR-219-5p overexpression cells. The expression of TBXT at mRNA level (**D**), and at protein level (**E**) in mock cells and in miR-219-5p overexpression cells. The expression of miR-219-5p (**F**) and TBXT (**G**) in miR-219-5p knockdown cells. The expression of miR-219-5p (**H**) and TBXT (**I**) in mammalian epithelium cells and breast cancer cells.

### miR-219-5p inhibits breast cancer cell EMT and migration and invasion through targeting TBXT

It has been reported that miR-219-5p inhibits breast cancer cell migration and EMT by targeting myocardin-related transcription factor A [31]. Because TBXT can function as an EMT inducer in several cancers [22–24], and we found that it is a novel target of miR-219-5p. We wondered whether the inhibition on EMT and cell migration and invasion by miR-219-5p in breast cancer cells were also mediated by TBXT. To assess the role of TBXT in this aspect, we ectopically expressed TBXT ORF in MDA-MB-231/miR-219-5p cells (Figure 2B). The three cell lines MDA-MB-231, MDA-MB-231/miR-219-5p and MDA-MB-231/miR-219-5p plus TBXT were used for this purpose. We first examined the cell viability of the three cell lines to get rid of the effect of cell death on EMT status and cell migration and invasion. We did not find any difference in cell viability among those cell lines (Figure 2A). Although we did not observe a clear morphological change in these cells (data not shown), we did observe obvious reduction in N-cadherin and vimentin level and acquired expression of E-cadherin in the cells that miR-219-5p is overexpressed (Figure 2C, middle panel). However, the re-introduction of TBXT in these cells counteracted the inhibition of miR-219-5p on EMT (Figure 2C, right panel). Similarly, the inhibition of miR-219-5p on cell migration and invasion is also rescued by re-expression of TBXT (Figure 2D,F). We also used miR-219-5p knockdown cell lines to perform migration and invasion assay and found that the migration and invasion capability of cells with low level miR-219-5p expression were significantly increased (Figure 2E,G). All these data suggest that miR-219-5p inhibits EMT and cell migration and invasion by targeting TBXT.

**Figure 2:** The inhibition on the breast cancer cell EMT and cell migration and invasion by miR-219-5p is mediated by TBXT (**A**) Cell viability of the three cell lines; MDA-MB-231 mock cells, MDA-MB-231 overexpressing miR-219-5p and MDA-MB-231 overexpressing miR-219-5p plus TBXT. (**B**,**C**) Immunoblotting of TBXT, E-cadherin, N-cadherin, vimentin in above three cell lines. Representative images and statistical results of Transwell migration assays (**D**) and Matrigel invasion assays (**F**) in the three cell lines. (**E**) Representative images and statistical results of Transwell migration assays and Matrigel invasion assays (**G**) of miR-219-5p knockdown cells and control cells. The data are presented as means ± SD of three independent experiments, and statistical significance was determined by two-tailed, unpaired Student’s *t* test. The quantification result shown on each graph represents the statistical analysis of three experiments.

### The inhibition of miR-219-5p on breast cancer cell migration and invasion is independent of hormone receptor and Her2 status

We have shown that miR-219-5p can significantly inhibit MDA-MB-231 cell migration and invasion (Figure 2D,F). MDA-MB-231 cell is a triple-negative breast cancer cell that does not have estrogen and progesterone receptors and does not overexpress HER2 protein. To prove the universal inhibition role of miR-219-5p on different type of breast cancer cells, we performed migration and invasion assays by using two additional breast cancer cell lines, MCF-7, that is estrogen and progesterone receptor positive and HER2 negative, and BT474, that expresses estrogen and progesterone receptor plus HER2 protein. Similar to its function in MDA-MB-231 cells, miR-219-5p dramatically inhibits migration and invasion of MCF-7 cells (Figure 3A) and BT474 cells (Figure 3B). This result indicated that the inhibition of miR-219-5p on breast cancer cell migration and invasion is not relevant to hormone receptor and HER2 signaling.

**Figure 3:** The inhibition of miR-219-5p on breast cancer cell migration andinvasion is not relevant to hormone receptor and Her2 status in cells (**A**) Representative images and statistical results of Transwell migration and Matrigel invasion assays of MCF-7 and MCF-7 overexpressing miR-219-5p cells. (**B**) Representative images and statistical results of Transwell migration and Matrigel invasion assays of BT474 and BT474 overexpressing miR-219-5p cells. The data are presented as means ± SD of three independent experiments, and statistical significance was determined by two-tailed, unpaired Student’s *t* test. The quantification result shown on each graph represents the statistical analysis of three experiments.

### The CSC features of MDA-MB-231 cells is diminished by miR-219-5p and is recovered by TBXT

Many reports have indicated that there is a possible link between cells going through EMT and cells with properties of CSCs [32]. Induction of EMT program can generate stem-like cells. Sarkar et al. reported that TBXT can confer colorectal cancer cells with CSC features [33]. Our results had shown that miR-219-5p inhibited EMT through its target TBXT, we wondered if miR-219-5p had any effects on regulating stem cell properties.

The stemness properties of CSCs are same as those of normal stem cells and can be identified by the pluripotency and self-renewal marker genes. The homeobox domain transcription factor Nanog is an important factor in regulating the pluripotency and self-renewal of embryonic stem cells. Nanog is reportedly expressed in human cancers and its expression has been frequently correlated with CSC marker expression [34]. Thus, we first checked if the expression of Nanog would be affected by miR-219-5p. TargetScan and miRBase analyses indicate that Nanog is not a target of miR-219-5p. As the results showed, overexpression of miR-219-5p in MDA-MB-231 cells did reduce the expression of Nanog either in transcription level (Figure 4A) or in translation level (Figure 4B, middle panel). However, the inhibition of miR-219-5p on Nanog expression can be offset by re-expression of TBXT in those cells (Figure 4A,B), which clearly demonstrating that miR-219-5p regulates CSC properties through its target TBXT. To further determine if miR-219-5p can change the CSC properties of MDA-MB-231 cells, we performed a qPCR assay for aldehyde dehydrogenase isoform 1 (*Aldh1*), a known marker for breast CSCs [35]. Our results showed that overexpression of miR-219-5p reduced the *Aldh1* level (Figure 4C). The effect of miR-219-5p on the properties of MDA-MB-231 CSCs was also examined by the mammosphere-forming capability of cells. The overexpression of miR-219-5p in MDA-MB-231 cells reduced the mammosphere-forming ability of cells, which can be recovered by re-expressing TBXT (Figure 4D).

**Figure 4:** miR-219-5p diminishes the CSC features of MDA-MB-231 cells (**A**) qPCR and (**B**) immunoblotting of Nanog in MDA-MB-231 mock cells, miR-219-5p overexpression MDA-MB-231 cells and miR-219-5p overexpression MDA-MB-231 that was introduced with TBXT. (**C**) qPCR of Aldh1 in the above three cell lines. (**D**) Quantification of mammosphere formation by the above three cell lines. The data are presented as means ± SD of three independent experiments, and statistical significance was determined by two-tailed, unpaired Student’s *t* test. The quantification result shown on each graph represents the statistical analysis of three experiments.

## Discussion

To date, many studies have proven that the dysregulation of miRNAs is associated with the initiation and development of human cancers. miRNAs can function not only as a tumor promoter but also as a tumor repressor. Either by silencing miRNA expression using antagomirs or expressing miRNA with its mimics, cellular miRNA can be controlled, which may be a novel potential therapeutic strategy. For example, researchers have found that silencing miR-10 can lead to the prevention of breast cancer metastasis [30], and overexpression of miR-26a was shown to suppress tumorigenesis in a murine liver cancer model [36].

The deficiency of miR-219-5p has been identified in colon cancer [37], gastric cancer [38], glioblastoma [39] and malignant melanoma [40]. miR-219-5p is up-regulated in hepatocellular carcinoma cells and overexpression of miR-219-5p confers the cells with high metastatic potential [41]. miR-219-5p functions as either an oncogene or a tumor suppressor depending the cellular context and the genes it targets. Our work showed that miR-291-5p can induce the re-appearance of E-cadherin, an epithelial cell marker, in mesenchymal MDA-MB-231 cells, and decrease the expression of N-cadherin and vimentin, two mesenchymal cell markers. Although miR-291-5p overexpression did not change the mesenchymal MDA-MB-231 cells to epithelial morphology, the expression alterations of these EMT marker genes strongly suggested miR-291-5p is an inhibitor of EMT. The expression changes of EMT marker genes are well-accepted indicator for EMT process happening. EMT is a complex process and has been shown to involve changes in the expression of ∼4000 genes [42]. miR-219-5p is one of EMT regulator, but may not be the master regulator. Although its overexpression can lead to EMT maker gene expression alternation, it may not be powerful enough to drive the mesenchymal cancer cell fully changing to epithelial morphology. Considering the complexity of EMT process and the regulation ability of an miRNA on multiple gene targets, it is understandable that miR-219-5p itself cannot completely drive mesenchymal–epithelial transition (MET), the reverse process of EMT. EMT is also characterized by cell motility and invasiveness change [43]. Our results found that overexpression of miR-219-5p inhibits cell migration and invasion, knockdown of endogenous miR-219-5p increases the cell ability to migrate and invade. These results are consistent with the reported role of miR-219-5p in breast cancer development [31].

In the present study, we identified TBXT as a novel target of miR-291-5p in breast cancer cells. TBXT is one member of the T-Box transcription factor family and is vital for the development of the vertebrate embryo [16]. Many reports have demonstrated that the expression of TBXT is higher in a variety of human carcinomas [20,21]. In human carcinomas, TBXT is able to regulate epithelial tumor plasticity by inducing epithelial tumor cells to undergo the EMT [22–24]. To verify whether miR-219-5p targeted TBXT, we cloned the 3′-UTR of TBXT into a luciferase reporter vector and performed a luciferase assay. The results confirmed that TBXT is a direct target of miR-219-5p. Subsequent rescue experiments have shown that re-expression of TBXT in miR-219-5p/MDA-MB-231 cells indeed reversed the inhibition of miR-219-5p on EMT and cell migration and invasion. Zhuang et al. found that miR-219-5p targets MRTF-A in breast cancer cells [31]. Our data indicate that TBXT is another novel miR-219-5p target, and in breast cancer cells, miR-291-5p can establish its inhibitory function on EMT and cell migration and cell invasion by targeting TBXT.

There is abundant evidence revealing a tight relationship between EMT process and the properties of CSCs [32]. TBXT has been found to be able to confer colorectal cancer cells with CSC features [33]. In agreement with these data, we found that after overexpressing miR-219-5p, the expression of two breast CSC markers, Nanog and ALDH1, was decreased. Furthermore, when re-expressing TBXT in miR-219-5p/MDA-MB-231 cells, the expression of these two marker genes was recovered to basal levels. The mammosphere formation experiment also confirmed that miR-219-5p affects the CSC features of MDA-MB-231 cells by targeting TBXT.

Taken together, we showed that TBXT is a novel target of miR-219-5p. By blocking the expression of TBXT, miR-291-5p acts as an inhibitor for EMT and migration and invasion of breast cancer cells. The elucidation of a new miR-219-5p/TBXT axis in breast cancer may provide a potential therapeutic strategy for cancer drug discovery in future.

## Data Availability

The data that support the findings of the present study are available from the corresponding author upon reasonable request.

## Abbreviations

CSC: cancer stem cell
EMT: epithelial–mesenchymal transition
miRNA: microRNA
ORF: open reading frame
qPCR: quantitative PCR
3′-UTR: 3′-untranslated region
